# In-Depth Study of *Thymus vulgaris* Essential Oil: Towards Understanding the Antibacterial Target Mechanism and Toxicological and Pharmacological Aspects

**DOI:** 10.1155/2022/3368883

**Published:** 2022-07-21

**Authors:** Sarra Akermi, Slim Smaoui, Mariam Fourati, Khaoula Elhadef, Moufida Chaari, Ahlem Chakchouk Mtibaa, Lotfi Mellouli

**Affiliations:** Laboratory of Microbial Biotechnology and Enzymes Engineering (LR15CBS06), Center of Biotechnology of Sfax (CBS), University of Sfax, Road of Sidi Mansour Km 6, P.O. Box 1177 Sfax 3018, Tunisia

## Abstract

Questions have been raised apropos the emerging problem of microbial resistance, which may pose a great hazard to the human health. Among biosafe compounds are essential oils which captured consumer draw due to their multifunctional properties compared to chemical medication drugs. Here, we examined the chemical profile and the mechanism(s) of action of the *Thymus vulgaris* essential oil (TVEO) against a Gram-negative bacterium *Salmonella enterica* Typhimurium ATTCC 10028 (*S. enterica* Typhimurium ATTCC 10028) and two Gram-positive bacteria *Staphyloccocus aureus* ATCC 6538 (*S. aureus* ATCC 6538) and *Listeria monocytogenes* ATCC 19117 (*L. monocytogenes* ATCC 19117). Findings showed that TVEO was principally composed of thymol, o-cymene, and *γ*-terpinene with 47.44, 16.55, and 7.80%, respectively. Molecular docking simulations stipulated that thymol and *β*-sesquiphellandrene (a minor compound at 1.37%) could target multiple bacterial pathways including topoisomerase II and DNA and RNA polymerases of the three tested bacteria. This result pointed plausible impairments of the pathogenic bacteria cell replication and transcription processes. Through computational approach, the VEGA quantitative structure–activity relationship (QSAR) model, we revealed that among twenty-six TVEO compounds, sixteen had no toxic effects and could be safe for human consumption as compared to the Food and Drug Administration (FDA) approved drugs (ciprofloxacin and rifamycin SV). Assessed by the SwissADME server, the pharmacokinetic profile of all identified TVEO compounds define their absorption, distribution, metabolism, and excretion (ADME) properties and were assessed. In order to predict their biological activity spectrum based on their chemical structure, all TVEO compounds were subjected to PASS (Prediction of Activity Spectra for Substances) online tool. Results indicated that the tested compounds could have multiple biological activities and various enzymatic targets. Findings of our study support that identified compounds of TVEO can be a safe and effective alternative to synthetic drugs and can easily combats hazardous multidrug-resistant bacteria.

## 1. Introduction

In recent years, antimicrobial-resistant (AMR) bacteria have been admitted as a public health risk that could cause an increase in the global burden of infectious disease [1–4]. For instance, each year, more than 670,000 infections and 700,000 deaths worldwide were provoked by AMR [5, 6]. Mutually controlled by host immune condition, microflora organization, and antimicrobial interventions, AMR evolution occurs with the multidrug resistance [7, 8]. While AMR could not be pragmatically eradicated, antimicrobials will endure to miss their potency, and, in the close future, more people may die from infections [9–11]. Therefore, it is crucial to explore original effective and broad-spectrum antibacterial agents to control bacteria, which can be antibiotic resistant, highly virulent, and high costs for the medication. Among the leading strategies for the exploration and detection of new targets in pathogens are the masterfully using bioinformatics tools. These tools can provide useful information for better comprehension of the interactions between targets and biomolecules and therefore help to anticipate new treatment targets for pathogenic microorganisms [12, 13].

Extracted from natural plants, essential oils (EOs) can be exploited as a practical alternative. More specifically, thyme (*Thymus vulgaris* L.), appertained to the family of *Lamiaceae* and the genus of *Thymus*, was consumed for centuries because of its medicinal properties and was generally recognized as safe (GRAS) by the FDA [14–17]. In addition, essential oil acquired from *Thymus vulgaris* L. had an extensive range of biological activities [17]. Thyme EO contains high levels of phenolic compounds, like thymol, carvacrol, p-cymene, and *γ*-terpinene [17, 18]. Interestingly, numerous studies reported that thymol, the major antibacterial component occurring in TEO, can destroy the bacterial cell membrane [19, 20]. Liu et al. revealed that thymol powerfully inhibit *Pseudomans aeruginosa* and directly change the cell structure [15]. *P*. *aeruginosa* cell membrane integrity is destroyed as evidenced by an increase in permeability of the inner/outer membranes. In other studies, Wang et al. and Lade et al. noted that thymol disrupts the *Staphylococcus aureus* membrane integrity to achieve the inner structure of the bacterial cell and joints to the minor groove of bacterial DNA, ensuring in a destabilization of the DNA secondary structure [21, 22].

In extension of our research to disclose the potential of natural therapeutic agents [13], this current investigation is aimed at elucidating the molecular docking interactions of all components of *Thymus* EO with bacterial DNA and RNA polymerases, as well as the topoisomerase II of *S. aureus*, *S. enterica* Typhimurium, and *L. monocytogenes* were profoundly reviewed *in silico*. As a part of our endeavor to increase the potential and exploration of these activities, a pharmacokinetics and computational toxicological studies were well discussed.

## 2. Materials and Methods

### 2.1. Plant Material, Essential Oil Extraction, and Gas Chromatography–Mass Spectrometry (GC–MS) Analysis

#### 2.1.1. Plant Material Collection and EO Extraction

*Thymus vulgaris* L. plant was collected from the region of Sfax, Tunisia (N: 34.4426°, E: 10.4537°) which is characterized by a semiarid climate. Aerial parts were harvested during the flowering stage in April 2022 and were air-dried in obscurity at room temperature. The EO of dried samples of *T. vulgaris* (TVEO) aerial parts was hydrodistilled for 3 h using a Clevenger apparatus.

#### 2.1.2. EO Analysis Using Gas Chromatography–Mass Spectrometry (GC–MS)

The analysis of TVEO was accomplished using a GC/MS HP model 6980 inert MSD, equipped with an Agilent Technologies capillary HP-5MS column (60 m × 0.25 mm, 0.25 mm film thickness) coupled to a mass selective detector (MSD5973, ionization voltage 70 eV, all Agilent, Santa Clara, CA, USA). The carrier gas was helium and has been maintained at 1.2 mL/min flow rate. The oven temperature program was as follows: 1 min at 100°C ramped from 100 to 280°C at 5°C/min and 25 min at 280°C. The chromatograph was equipped with a split/split less injector used in the split less mode. Identification of TVEO components was achieved by matching their mass spectra with Wiley Registry of Mass Spectral Data 7th edition (Agilent Technologies) and National Institute of Standards and Technology 05 MS (NIST) library data.

### 2.2. Antibacterial Activity

#### 2.2.1. Microorganisms and Growth Conditions

In order to evaluate TVEO antibacterial activity, two Gram-positive bacteria: *S. aureus* ATCC 6538 and *L*. *monocytogenes* ATCC 19117, and two Gram-negative bacteria: *S. enterica* Typhimurium ATCC 14028 and *E. coli* ATCC 8739, were selected. Bacterial cultures were deposited in 3 mL of Luria-Bertani (LB) agar medium composed of (g/L): peptone, 10; yeast extract, 5; NaCl, 5; and agar, 20 at pH 7.2; then, the bacterial strains were incubated at 37°C according to the method described by [23].

#### 2.2.2. Agar Diffusion Method

Antimicrobial activity of TVEO was evaluated by agar-well diffusion assay according to a method proposed by Güven et al. [24]. Fifteen milliliters of the molten agar (45°C) were flowed into sterile Petri dishes (*Ø* 90 mm). Bacterial cell suspensions were prepared, and 100 *μ*L was evenly deposited onto the surface of plates containing LB agar medium. Plates were aseptically dried, and then, 5 mm wells were punched into the agar with a sterile Pasteur pipette. TVEO was dissolved in DMSO, water (1/9; *v*/*v*) to a final concentration of 1 mg/mL and then filtered through 0.22 *μ*m pore size black polycarbonate filters. 100 *μ*L of this filtered solution was placed into each well, and the plates were incubated at 37°C. Gentamicin (10 *μ*g/wells) was used as a positive control.

#### 2.2.3. Minimal Inhibitory Concentration (MIC)

MIC is defined as the lowest concentration that could inhibit the visible growth of the tested microorganism. In this context, MIC of TVEO was tested against four pathogenic bacteria which are as follows: two Gram-positive bacteria: *S. aureus* ATCC 6538 and *L*. *monocytogenes* ATCC 19117, and two Gram-negative bacteria: *S. enterica* Typhimurium ATCC 14028 and *E. coli* ATCC 8739, using the microdilution method with serial dilution described by Chandrasekaran and Venkatesalu [25]. Then, bacterial suspension was added with a final inoculum concentration of 10^6^ CF/mL. The contents of the tubes were mixed by pipetting and were incubated for 24 h at 37°C. For the antibacterial activity determination (inhibition zones and CMIs), each experiment was carried out simultaneously in triplicate under same conditions. The obtained diameters of inhibition zones were measured in mm and the MIC values were reported in mg/mL.

### 2.3. Interaction Study between TVEO Compounds and Selected Bacterial Targets by Molecular Docking

Receptor targets Fasta sequences of *S. aureus* ATCC 700699, *S. enterica* Typhimurium ATCC 700720, and L. *monocytogenes* ATCC 19115 were obtained from UniProt database [26] and NCBI database [27]. Protein models were projected to SWISS-MODEL server [28] for molecular homology modeling approach [29]. Validation of the obtained models was performed by checking Ramachandran plots and the QMEAN values [30], using PROCHECK analysis tool integrated in Profunc server ([31]. SMILES (simplified molecular input line entry systems) strings of TVEO compounds were obtained from the PubChem database [32] and controls (rifamycin SV and ciprofloxacin). SMILES structures were downloaded from the DrugBank database [33], and all were converted into 3D structure using CORINA demo webserver [34] and then saved in pdb file format. Molecular docking was performed using the AutoDock Vina software (version 1.2.0) to calculate free energy of binding (kcal/mol) scores according to the methodology proposed by [35]. The docking position results were visualized using Discovery Studio version 16.1.0 (Dassault Systemes BIOVIA, 2016).

### 2.4. Toxicity Prediction of Compounds by VEGA HUB Software Using QSAR Method

All TVEO compounds and the two controls (rifamycin SV and ciprofloxacin) were subjected to 8 toxicity measurements in a view to assess carcinogenicity, mutagenicity, developmental/reproductive toxicity, endocrine disrupting ability, and genotoxicity. All tests were performed by VEGA software version 1.1.5 using the QSAR (quantitative structure–activity relationship) approach [36].

### 2.5. ADME Analysis

Pharmacokinetics, drug-likeness, and medicinal chemistry properties of TVEO compounds were predicted using SwissADME which is an open access software for ADME parameters evaluation and profiling [37].

### 2.6. *In Silico* Prediction of Possible Bioactivities

The PASS software was used to predict bioactivity of molecules based on the structural similarity to the large data base of known active substances in order to find new TVEO molecule targets [38, 39].

### 2.7. Statistical Analysis

All tests were assayed in triplicate and expressed as the mean ± standard deviation of the measurements. The statistical program SPSS version 21.00 for Windows (SPSS Inc., Chicago, IL, USA) was used to analyze the data. Variance was analyzed by one-way ANOVA and Student's *t*-test was applied to compare each parameter at *p* < 0.05.

## 3. Results and Discussion

### 3.1. Chemical Composition Analysis of TVEO

GC-MS analysis of TVEO revealed the existence of 26 different components (Table 1). The main components were thymol, the most abundant compound (47.44%), followed by o-cymene (16.55%), *γ*-terpinene (7.80%), and linalool (4.41%). Moreover, it detected the presence of 4 compounds which their percentages (EO %) were more than 2%. These later are the *α*-zingibirene (3.40%), *β*-myrcene (2.36%), caryophyllene (2.09%), and borneol (2.02%).

Thymol, known also by the chemical name 2-isopropyl-5-methylphenol, is a natural phenol monoterpene [40] importantly detected in *Lamiacaeae* family [41] including many plant species such as *Thymus vulgaris L.* [42], *Ocimum gratissimum L.* [43], *Origanum L*. [44], and *Trachyspermum ammi L.* [45] and other species of the genus *Satureja L*. [46] and *Monarda L.* [47]. This volatile monoterpenoid is largely used by nutraceutical, pharmaceutical, and cosmeceutical industries due to its multiple potential therapeutic properties [48–58]. In addition, thymol was globally recognized-as-safe food additive according to US department of Food and Drug Administration (FDA) [59].

O-cymene, known as 1-isopropyl-2-methylbenzene, is an acyclic monoterpene which belongs to p-cymene isomers and has an orthosubstituted alkyle group [60]. Previous studies demonstrated that o-cimene has several therapeutic effects [61–66]. Several studies indicated the existence of a remarkable synergetic effect between ocimene and other terpenes such as *α*-pinene and myrcene which were noticed to produce more beneficial effects when combined [67, 68].

*γ*-Terpinene, renowned also as p-mentha-1,4-diene, is a naturally occurring monoterpene hydrocarbon [69] that has been isolated from many botanical sources including *Origanum vulgare*, *Citrus limon* L*, Melaleuca alternifolia*, and *Eucalyptus obliqua* [70, 71]. This monoterpene is largely employed in food, cosmetics, and pharmaceutical industries [72]. Previous research showed that *γ*-terpinene has potential biological activities such as antioxidant [73], anti-inflammatory [74], and antimicrobial activities [75, 76].

On the other hand, linalool, known as 3,7-dimethyl-1,6-octadien-3-ol [77], is a naturally occurring acyclic monoterpenoid and tertiary alcohol which is commonly found as a major active component in the essential oil of several aromatic plant species [78] principally in *Lamiaceae* and *Lauraceae* botanical families. It has been reported that this monoterpenol is broadly used in food industry as an aromatic and preservative agent, in cosmetic as a fragrance and antiseptic constituent [79–83].

It should be noted that TVEO composition may depend on many biotic and abiotic factors including seasonal variations of temperature and humidity [84], phenological stages and different vegetation cycles [85], geographic location [86], environmental stress [87], and extraction technique [88]. Aljabeili et al. reported that the TVEO collected from KSA showed a significant composition variation and the major compounds were thymol (41.04%), 1,8-cineole (14.26%), *γ*-terpinene (12.06%), and p-cymene (10.50%) [89]. Another study revealed that Turkish TVEO has different components amounts such as thymol (49%), *β*-cymene (19.99%), carvacrol (7.63%), and *trans*-caryophyllene (6.79%) [90]. In addition, Moghaddam et al. reported that Iranian TVEO contains thymol (36.81%), *ρ*-cymene (30.90%), and carvacrol (3.16%) [91].

### 3.2. Antibacterial Activity

As represented in Table 2, TVEO displayed an interesting antibacterial activity against the four tested bacterial strains with inhibition zones ranging from of 21 to 23 mm against Gram-negative and Gram-positive bacteria, respectively. In addition, it is important to note that monoterpenes exhibit a broad-spectrum antibacterial activity against pathogenic bacteria [92, 93]. This fact could be explained by the presence of a lipophilic character which provides to monoterpenes the ability to adhere to bacterial cell membrane lipids and to deploy their antibacterial action [94]. In our study, the obtained MIC values mentioned in Table 2, indicated that TVEO was more potent (*p* < 0.05) against Gram-positive bacteria (MICs = 0.097 mg/mL) than Gram-negative bacteria (MICs = 0.195 mg/mL). These findings were in agreement with previous studies which reported that Gram-positive bacteria are susceptible to be more sensitive to plant EOs than Gram-negative bacteria due to the existence of lipopolysaccharides which acts as a hydrophobic barrier [95, 96].

### 3.3. Interactions between TVEO Molecules and Bacterial Topoisomerase II and DNA and RNA Polymerases

Computational modeling is a 3R-based approach and an attractive alternative to experiments in a view to understand bioactive compounds mechanism of action and their antibacterial inhibitory process [97]. Molecular docking was performed to predict different TVEO components that could bind specifically to select bacterial receptors active sites responsible for DNA replication and transcription processes. In this respect, we investigated TVEO antibacterial inhibitory effect on topoisomerase II (DNA gyrase) and DNA and RNA polymerases of three pathogenic bacteria *S. aureus* ATCC 700699, *S. enterica* Typhimurium ATCC 700720, and *L*. *monocytogenes* ATCC 19115. Molecular homology results indicated that selected templates can be used for molecular modeling (Table 3); their identities (%) are higher than 30% [98], and Ramachandran plot values of favored regions and allowed regions were over 90% [99].

Moreover, it is necessary to remind that DNA and RNA polymerases are crucial enzymes involved in the DNA replication, transcription, and translation as well as nucleic acid formation in bacterial cells [100]. On the other hand, topoisomerase II (DNA gyrase) is also implicated in DNA replication and transcription processes and has an imperative role characterized by its ability to catalyze the unwinding of supercoiled DNA strands [101]. These imperative enzymes constitute attractive and validated targets for antibacterial agents [102]. Molecular docking simulation results are elucidated by (Table 4). These later displayed that TVEO major compound thymol (47.44%) showed a good inhibitory effect on topoisomerase II, RNA polymerase, and DNA polymerase of the selected pathogenic bacteria.

A previous study conducted by Liu et al. reported that thymol has a potential antibacterial activity against *P*. *aeruginosa* [15]. This monoterpenoid can affect bacterial DNA normal function. It could block gene expression processes including replication, transcription, and expression by intercalation with bacterial DNA leading to bacterial death. The same study indicated that thymol could destroy bacterial membrane integrity by affecting its permeability and it could also hinder biofilm formation. Another research paper displayed that thymol could bind to bacterial DNA, modulate its structure, and prohibit its biological function [103]. Furthermore, dos Santos Barbosa et al. showed that the antibacterial inhibitory activity of *Origanum vulgare* EO was effective against *Salmonella Enteritidis* due to the presence of thymol which caused interference in protein regulation as well as DNA synthesis [104]. On the other hand, the minor compound *β*-sesquiphellandrene (1.34%) showed the lowest free energy of binding (Kcal/mol) and the highest inhibitory potential on topoisomerase II and DNA and RNA polymerases of the selected pathogenic bacteria (Table 4). A previous study reported that *β*-sesquiphellandrene was responsible for the high antibacterial and antioxidant activities of some pomelo varieties' EOs [105]. Another study indicated that the presence of *β*-sesquiphellandrene presented in ginger (*Zingiber officinale*) essential oil could make this later as a potential antimicrobial agent by inhibiting mycobacterial acyl carrier protein reductase enzyme and Enoyl acyl carrier protein reductase activities [106].

A recent study showed that *Cupressus sempervirens* EO had a great inhibitory effect on DNA gyrase and DNA and RNA polymerases of *S. aureus* and *S. enterica* owing to the presence of *α*-pinene, *δ*-3 carene, and borneol [13]. Moreover, a previous study conducted by [107] evaluated the inhibitory effect of *Litsea cubeba* EO on topoisomerase and DNA and RNA polymerases of *E.coli.* Another study revealed that the germacrene B, a minor compound in *Siparuna guianensis* EO, had an effective inhibitory activity against bacterial DNA and RNA polymerases of multiple pathogenic bacteria including *E.coli*, *P. aeruginosa*, *S. aureus*, and *S. pyogenes* [108]. Therefore, these findings confirmed that TVEO has a powerful inhibitory effect on pathogenic bacteria based on the inhibition of DNA replication and transcription processes. Consequently, we project in subsequent work to perform further in vitro assays based on the evaluation of protein-molecule binding assays.

Interaction profiles details of thymol and *β*-sesquiphellandrene with the active sites of the selected targets of *S. aureus* ATCC 700699, *S. enterica* Typhimurium ATCC 700720, and *L. monocytogenes* ATCC 19115 are summarized in Table 5.

Interaction profile results of thymol and *β*-sesquiphellandrene with topoisomerase II and DNA and RNA polymerases of *S. aureus* are presented by Figures 1 and 2. Thymol made a complex with DNA polymerase receptor via alkyl interaction and conventional hydrogen bond with LYS228 and van der Waals interactions with ASN84, LYS88, LEU87, GLU469, TYR91, LEU227, and ILE492 (Figure 1(a)). Additionally, RNA polymerase complexed with thymol had alkyl and Pi-alkyl interaction with VAL536 and LYS35; van der Waals interactions with GLU413, SER410, GLY412, SER36, and GLU538; and Pi-sigma interaction with TRP39 (Figure 1(b)). Likewise, it interacted with topoisomerase II via alkyl interaction with ALA614; van der Waals interactions with HIS46, ARG198, TRP49, ARG42, THR194, GLN197, THR617, and LEU608; and two conventional hydrogen bonds with ASP610 and GLU609 (Figure 1(c)).

*β*-Sesquiphellandrene complexed with DNA polymerase showed Pi-alkyl interaction with LEU641 and van der Waals interactions with ILE938, LYS901, PHE900, ASP936, GLU939, ILE899, SER903, LEU902, and GLN975 (Figure 2(a)). When complexed with RNA polymerase, it made Pi-alkyl interaction with VAL270, LYS35, and VAL536; van der Waals interactions with SER36, SER410, GLY412, ARG407, GLN416, GLN413, GLU538, and ILE32; and Pi-sigma interaction with TRP39 (Figure 2(b)). Concerning topoisomerase II, *β*-sesquiphellandrene displayed alkyl and Pi-alkyl interactions with VAL606, PHE618, ILE532, ALA614, LEU521, and LEU608 and van der Waals interactions with LYS607, ARG198, GLU609, GLU613, ASP610, and TYR525 (Figure 2(c)).

On the other hand, interaction profiles between thymol and *β*-sesquiphellandrene with topoisomerase II and DNA and RNA polymerases of *S*. e*nterica* Typhimurium are outlined in Figures 3 and 4. DNA polymerase complexed with thymol showed alkyl and Pi-alkyl interactions with ARG18 and LYS17 and van der Waals interactions with ASP1188, THR657, SER656, PRO19, ASN622, ASN620, SER621, LEU623, and ALA 619 (Figure 3(a)). Thymol complex with RNA polymerase indicated the presence of alkyl interaction with MET768 and van der Waals interactions with ASP785, GLN767, ASN766, GLY786, PRO787, SER788, PRO691, THR692, ALA695, THR789, and LEU693 (Figure 3(b)). This monoterpene also made interactions with topoisomerase II via alkyl interactions with VAL727, ILE557, and ALA560; van der Waals interactions with LEU561, VAL584, LEU723, GLN591, and ASP553; and one conventional hydrogen bond with ASN588 (Figure 3(c)).

The complex of *β*-sesquiphellandrene and the DNA polymerase of *S. enterica* Typhimurium revealed the existence of alkyl and Pi-akyl interactions with LEU75, ALA94, LEU129, LEU32, PHE35, and ILE39 and van der Waals interactions with GLN41, GLN36, GLY76, and MET130 (Figure 4(a)). This sesquiterpene complexed with RNA polymerase showed alkyl and Pi-alkyl interactions with MET130, LEU32, LEU129, PHE35, ALA94, and LEU75 and van der Waals interactions with ILE39, GLN36, and ASP32 (Figure 4(b)). In addition, it made interactions with topoisomerase II via alkyl and Pi alkyl interactions with VAL467, PHE513, PHE777, ARG516, and LEU462 and van der Waals interactions with MET461, LEU509, and THR512 (Figure 4(c)).

DNA polymerase receptor of *L. monocytogenes* complexed with thymol displayed the existence of alkyl and Pi-alkyl interactions with MET389, LEU345, LEU394, ILE392, and PHE367 and van der Waals interactions with GLU359, THR357, LYS358, ILE343, THR360, and SER364 (Figure 5(a)). It also showed when complexed with RNA polymerase alkyl interactions with LYS283 and LYS284 and van der Waals interactions with VAL150, GLY149, TYR151, ASN410, ASP403, ASP571, and ASN289 (Figure 5(b)). Further, thymol made interactions with topoisomerase II via alkyl interaction with PHE97; van der Waals interactions with GLN95, SER98, GLN267, TYR266, THR220, VAL268, ASN269, GLY115, and SER112; and one conventional hydrogen bond with VAL113 (Figure 5(c)).

Finally, *β*-sesquiphellandrene complex with DNA polymerase of *L. monocytogenes* indicated the existence of Alkyl interactions with MET386, ALA382, ILE399, and LEU488 and van der Waals interactions with SER397, PHE492, PRO489, GLU484, THR400, and THR491 (Figure 6(a)). It showed also with RNA polymerase alkyl interactions with LYS280, LYS284, and TYR151 and van der Waals interactions with VAL150, GLY149, ASP403, ASN410, ASP571, ASP404, ASP401, ASN289, and LYS283 (Figure 6(b)). In addition, *β*-sesquiphellandrene made a complex with topoisomerase II via alkyl and Pi-alkyl interactions with VAL113, ILE264, and PHE97 and van der Waals interactions with GLY115, SER112, GLN95, ARG92, GLY111, PHE88, SER98, ASN269, VAL268, THR220, PRO265, and TYR266 (Figure 6(c)).

### 3.4. *In Silico* TVEO Compound Toxicity Evaluation by VEGA QSAR Model

Toxicity evaluation of different TVEO compounds and the two selected FDA-approved antibiotics, used as controls (rifamycin SV and ciprofloxacin), was performed by the help of QSAR (quantitative structure–activity relationship) approach and using VEGA HUB software. We chose to assess compounds toxicity based on 8 different toxicity measurements. Results are represented by (Table 6) and revealed that FDA-approved drugs could be toxic in several assays. In this context, rifamycin SV and ciprofloxacin are found to be mutagenic in the mutagenicity test/model (Ames test) and predicted to engender developmental/reproductive toxicity. These two antibiotics were also predicted to be genotoxic according to the in vitro micronucleus activity model. However, many TVEO compounds such as *α*-pinene, *α*-thujene, camphene, *β*-pinene, 3-carene, D-limonene, *γ*-terpinene, terpinolene, linalool, borneol, 4-terpineol, *α*-terpineol, thymol, caryophyllene, *α*-bisabolene, and *β*-sesquiphellandrene showed nontoxic effects. Computational toxicity results confirmed that TVEO molecules could be used as a safe antimicrobial agents and economically low-cost alternative as compared to synthetic antibiotics. It is important to mention that research related to toxicological profiles of different essential oil compounds are poorly studied due to experiments complexity, expensive cost, and difficulty to detect toxicity variation because of the chemical function and factor variability [109]. However, previous studies indicated that toxicity is a dose-/concentration-dependent manner and thymol could have a certain limit of toxicity ranging from 36 mg/mL to 49 mg/mL with less risks of accumulation in body tissues and suggested to replace synthetic drugs, which has more side effect [110]. In addition, Schönknecht et al. confirmed the safety and the effectiveness of the drug containing the extracts of thyme with the addition of thymol (Bronchosol®) in cough treatment instead of using the synthetic drug ambroxol [111]. Concerning *β*-sesquiphellandrene, it was reported that this sesquiterpenoid could have a great anticancer activity and can be safe to use as compared to synthetic chemotherapeutic agents velcade, thalidomide, and capecitabine [112]. Nevertheless, more toxicological *in vitro*/*in vivo* data are needed to validate the safety of these phytochemicals. Thus, computational toxicity assessment could be the best alternative that would give robust data, avoid unnecessary waste of reagents, and minimize cruelty and sacrifices of lab animal testing.

### 3.5. TVEO Component ADME Analysis

In the present study, SwissADME server was used to determine some pharmacokinetics parameters included in absorption, distribution, metabolism, and excretion (ADME), drug-likeness, and medicinal chemistry characteristics for all TVEO compounds as represented in (Table 7). Results revealed that all TVEO components possess slow passive gastrointestinal absorption (GI) except linalool, camphor, borneol, 4-terpineol, *α*-terpineol, thymol methyl ether, and thymol which were predicted to have high GI permeability. Additionally, only sesquiterpenes including caryophyllene, *α*-humulene, *α*-amorphene, *α*-curcumene, *α*-zingibirene, *α*-bisabolene, and *β*-sesquiphellandrene were found not to be blood-brain barrier (BBB) permanent due to their heavy molecular weight. However, rest of compounds could easily cross the blood-brain barrier for that reason it could be suggested as potent central nervous system antioxidants and effective drug candidates in the treatment of neurodegenerative diseases like Alzheimer's and Parkinson's [113]. On the other part, none of the tested compounds was predicted to be P-gp transporter substrate. Concerning Cytochrome p450 (CYP) isoenzymes which are involved in 50-90% of therapeutic molecules biotransformation processes in a view to reduce metabolites accumulation in blood/tissues and drug-drug interaction risks [114], thymol methyl ether and thymol were predicted to be CYP1A2 inhibitors. Many TVEO molecules were predicted to inhibit CYP2C9 and CYP2D6 inhibitors. However, none of the compounds showed an inhibitory effect towards the CYP3A4. Moreover, skin permeation coefficient (log Kp) indicated that all compounds were impermeable through the skin barrier. Interestingly, TVEO drug-likeness score was acceptable with good bioavailability score (>10%) and the absence of violations related to known rules such as Lipinski's rule of five that predicts drug permeability and absorption based on H-bond donors, H-bond acceptors, molecular weight (MW > 500), and a calculated log *p*) [115], as well as Veber. Both rules are a mainstay of decision-making in drug design and development and in the present study; both were validated. Furthermore, medicinal chemistry parameters revealed that none of the selected molecules returns any pan-assay interference compounds (PAINS) alert. The synthetic accessibility values of TVEO compounds indicated that these later could be synthesized for pharmaceutical uses.

### 3.6. Prediction of Possible Activity Spectra of TVEO Components

All TVEO compounds were subjected to PASS (Prediction of Activity Spectra for Substances) online tool intending to predict their biological activity spectrum based on their chemical structure. Results indicated that the tested compounds could have multiple biological activities and various enzymatic targets (Table 8). We have selected the top three activities which showed a Pa ≥ 0.7. Pa and Pi values indicated the probability of the selected molecule to be active/ inactive towards the targeted receptor. Mojumdar et al. reported that the probability of experimental pharmacological action is high when Pa > 0.7; however, the chance of finding the activity experimentally is less when Pa < 0.5 [116]. Interestingly, TVEO major compounds such as thymol which were predicted, in earlier section by molecular docking, to have a potent antibacterial activity on pathogenic bacteria by inhibiting DNA replication and transcription processes, displayed the existence of other biological activities including the ability to inhibit bacterial membrane permeability (Pa = 0.876) and it was anticipated to enhance AP0A1 expression (Pa = 0.830) involved in the cellular synthesis of beneficial HDL [117]. In addition, O-cymene was predicted to be mitochondria ubiquinol-cytochrome-c reductase inhibitor (Pa = 0.924) (antifungal activity), mucomembranous protector (Pa = 0.842), and a fibrinolytic agent (Pa = 0.778) which could stimulate the dissolution of blood clots. Concerning *γ*-terpinene, it was predicted to treat skin eczema (Pa = 0.854) and phobic disorders (Pa = 0.803) owing to its ability to cross the blood-brain barrier (BBB). Finally, PASS prediction revealed that the minor compound *β*-sesquiphellandrene has other possible biological activities including antineoplastic effect (Pa = 0.827) and antipsoriatic (Pa = 0.750) and could be also used as immunosuppressant agent during organ transplant (Pa = 0.702) instead of using synthetic compounds such as cyclosporin A which was demonstrated to cause severe cholestatic liver disease [118]. These findings could provide more insights towards further in vivo and in vitro assays to validate the computational predictions.

## 4. Conclusion

The dramatical increase of antibiotic resistance urged scientists to diverge towards the use of aromatic medicinal plants essential oils to tackle the spread of superbugs. In that regard, the present study is aimed at investigating the TVEO chemical composition and antibacterial mechanism of action against *S. aureus* ATCC 6538, *S. enterica* Typhimurium ATCC 14028, and *L. monocytogenes* ATCC 19117. In addition, chemocomputational toxicological profile and pharmacological proprieties were developed. Interestingly, molecular docking simulations revealed that TVEO compounds such as thymol and *β*-sesquiphellandrene had an effective antibacterial activity against the tested bacteria by inhibiting topoisomerase II and DNA and RNA polymerase functions leading to vigorous impairment of bacterial DNA replication and transcription processes. Additionally, through VEGA QSAR, we demonstrated that TVEO could be a safe resource for potential antibacterial agents. Moreover, ADME analysis showed that both compounds fulfill the Lipinski's rule of five and could be used as potential candidate to overcome antibiotic resistance. Likewise, the *in silico* PASS prediction studies disclosed the presence of other useful bioactivities and possible enzymatic targets of TVEO which would be applied in the future to reduce the impact of several lethal diseases.

## Figures and Tables

**Figure 1:** Thymol complexed with DNA polymerase (a), RNA polymerase (b), and topoisomerase II (c) of *S. aureus.*

**Figure 2:** *β*-Sesquiphellandrene complexed with DNA polymerase (a), RNA polymerase (b), and topoisomerase II (c) of *S. aureus.*

**Figure 3:** Thymol complexed with DNA polymerase (a), RNA polymerase (b), and topoisomerase II (c) of *S. enterica* Typhimurium.

**Figure 4:** *β*-Sesquiphellandrene complexed with DNA polymerase (a), RNA polymerase (b), and topoisomerase II (c) of *S. enterica* Typhimurium.

**Figure 5:** Thymol complexed with DNA polymerase (a), RNA polymerase (b), and topoisomerase II (c) of *L. monocytogenes.*

**Figure 6:** *β*-Sesquiphellandrene complexed with DNA polymerase (a), RNA polymerase (b), and topoisomerase II (c) of *L. monocytogenes.*

**Table 1:** Chemical composition of TVEO.

Compound	Molar mass (g/mol)	Molecular formula	Retention time (min)	EO (%)
*α*-Pinene	136.23	C_10_H_16_	5.99	1.74
*α*-Thujene	136.23	C_10_H_16_	6.15	1.61
Camphene	136.23	C_10_H_16_	6.66	1.60
*β*-Pinene	136.23	C_10_H_16_	7.39	0.29
*β*-Myrcene	136.23	C_10_H_16_	7.85	2.36
*α*-Fellandrene	136.23	C_10_H_16_	8.17	0.34
3-Carene	136.23	C_10_H_16_	8.31	0.16
D-Limonene	136.23	C_10_H_16_	8.52	1.61
O-Cymene	134.22	C_10_H_14_	8.88	16.55
Cymol	134.22	C_10_H_14_	9.46	0.09
*γ*-Terpinene	136.23	C_10_H_16_	9.79	7.80
Terpinolene	136.23	C_10_H_16_	10.56	0.10
Linalool	154.25	C_10_H_18_O	11.03	4.41
Camphor	152.23	C_10_H_16_O	12.14	1.15
Borneol	152.23	C_10_H_18_O	12.84	2.02
4-Terpinenol	152.23	C_10_H_18_O	13.23	0.92
*α*-Terpineol	152.23	C_10_H_18_O	13.90	0.10
Thymol methyl ether	164.24	C_11_H_16_O	14.99	0.43
Thymol	150.22	C_10_H_14_O	16.48	47.44
Caryophyllene	204.35	C_15_H_24_	19.59	2.09
*α*-Humulene	204.35	C_15_H_24_	20.43	0.03
*α*-Amorphene	204.35	C_15_H_24_	20.99	0.10
*α*-Curcumene	202.33	C_15_H_22_	21.17	0.71
*α*-Zingibirene	204.35	C_15_H_24_	21.49	3.40
*α*-Bisabolene	204.35	C_15_H_24_	21.79	1.12
*β*-Sesquiphellandrene	204.35	C_15_H_24_	22.17	1.34
Monoterpenes hydrocarbons				34.25%
Oxygenated monoterpenes				56.47%
Sesquiterpens				8.79%
Total				99.51%

**Table 2:** Antibacterial activity of TVEO and the control gentamicin. Zones of growth inhibition was expressed in mm, and minimum inhibitory concentrations (MICs) were expressed in mg/mL.

Bacterial strains	Inhibition zone diameters (mm)		MIC (mg/mL)	
	TVEO	Gentamicin	TVEO	Gentamicin
*S. aureus* ATCC 6538	23 ± 1.00^b^	20 ± 0.83^a^	0.097 ± 0.00^b^	0.013 ± 0.00^b^
*L. monocytogenes* ATCCC 19117	22 ± 1.00^b^	20 ± 0.75^a^	0.097 ± 0.00^b^	0.013 ± 0.00^b^
*S. enterica* Typhimurium ATCC 14028	23 ± 1.00^a^	25 ± 1.25^b^	0.097 ± 0.00^b^	0.005 ± 0.00^b^
*E. coli* ATCC 8739	21 ± 0.83^a^	25 ± 1.25^b^	0.195 ± 0.00^b^	0.005 ± 0.00^b^

A Student *t*-test was used to determine the significant differences between inhibition zones and MIC.

**Table 3:** Receptors models of the selected pathogenic bacteria used in molecular docking simulation with TVEO constituents.

Bacterial Strain	Bacterial Target	Receptor	Template	Identity (%)	Ramachandran Plot		QMEAN
					Favored regions (%)	Additional allowed regions (%)	
*S. aureus* ATCC 700699	DNA polymerase	P63979 (UniProt)	4IQJ.1.L	36.77	87.9	10.1	−3.26
	RNA polymerase	Q932F8 (UniProt)	6WVK.1.C	81.09	85.5	12.7	−2.36
	Topoisomerase II	P66936 (UniProt)	6GAV.1.A	54.42	88.4	10.7	−1.69
*S. enterica* Typhimurium ATCC 700720	DNA polymerase	P14567 (UniProt)	5FKU.1.A	96.72	88.0	10.0	−2.35
	RNA polymerase	P06173 (UniProt)	4LLG.2.C	98.66	88.0	11.0	−1.11
	Topoisomerase II	P0A213 (UniProt)	4TMA.2.B	95.41	90.2	9.2	−1.82
*L. monocytogenes* ATCC 19115	DNA polymerase	WP031669548 (NCBI)	6VDE.1.A	38.30	81.6	16.4	-3.91
	RNA polymerase	GAT39567 (NCBI)	6WVK.1.C	86.10	87.1	11.4	-2.24
	Topoisomerase II	GAT39106 (NCBI)	2XCR.2.A	69.59	87.4	10.4	-2.01

**Table 4:** Molecular docking results for complexes of *T. vulgaris* EO compounds against DNA and DNA polymerases of *S. aureus* ATCC 700699, *S. enterica* Typhimurium ATCC 700720, and *L. monocytogenes* ATCC 19115 using Autodock Vina (kcal/mol).

Bacterial target	*S. aureus* ATCC 700699			*S. enterica* Typhimurium ATCC 700720			*L.monocytogenes* ATCC 19115		
Compound	DNA polymerase	RNA polymerase	Topoisomerase II	DNA polymerase	RNA polymerase	Topoisomerase II	DNA polymerase	RNA polymerase	Topoisomerase II
*α*-Pinene	-5.1	-6.1	-5.3	-5.4	-5.4	-5.2	-5.9	-6.0	-5.4
*α*-Thujene	-4.9	-5.4	-5.5	-5.3	-5.2	-5.3	-5.5	-5.3	-5.6
Camphene	-5.2	-6.0	-5.6	-5.2	-5.2	-5.0	-6.1	-5.9	-5.3
*β*-Pinene	-5.2	-5.7	-5.2	-5.5	-5.7	-5.3	-5.9	-6.0	-5.2
*β*-Myrcene	-4.9	-5.0	-5.2	-5.1	-5.1	-5.0	-5.2	-5.0	-5.0
*α*-Fellandrene	-5.2	-5.6	-5.4	-5.1	-5.1	-5.1	-5.5	-5.5	-5.6
3-Carene	-5.2	-5.6	-5.2	-5.6	-5.6	-5.5	-5.6	-5.5	-5.7
D-Limonene	-5.1	-6.0	-5.4	-5.4	-5.4	-5.1	-5.5	-5.6	-5.6
O-Cymene	-5.3	-5.5	-5.6	-5.7	-5.4	-5.4	-5.8	-5.5	-5.5
Cymol	-5.2	-5.7	-5.6	-5.5	-5.5	-5.2	-6.0	-5.9	-5.7
*γ*-Terpinene	-5.3	-6.0	-5.6	-5.8	-5.6	-5.7	-5.8	-5.8	-5.6
Terpinolene	-5.4	-5.8	-5.6	-5.6	-6.0	-5.6	-5.8	-5.6	-5.8
Linalool	-5.0	-5.2	-5.2	-5.5	-5.6	-5.4	-5.8	-5.1	-5.2
Camphor	-5.3	-6.0	-5.4	-5.4	-5.2	-5.3	-6.0	-5.6	-5.2
Linderol (borneol)	-5.4	-5.7	-5.5	-5.3	-5.3	-5.2	-5.8	-5.7	-5.3
4-Terpineol	-5.4	-6.2	-5.8	-5.8	-5.8	-5.5	-5.9	-6.0	-5.8
*α*-Terpineol	-5.4	-6.0	-5.6	-5.6	-5.8	-5.0	-5.8	-5.6	-5.8
Thymol methyl ether	-5.5	-5.8	-5.6	-5.3	-5.4	-4.9	-5.6	-5.5	-5.7
Thymol	-6.3	-6.2	-6.6	-6.4	-6.6	-6.2	-6.8	-6.7	-6.6
Caryophyllene	-6.0	-6.4	-6.7	-6.4	-6.5	-6.4	-6.5	-6.3	-6.4
*α*-Humulene	-6.3	-6.3	-6.9	-6.4	-7.1	-6.1	-6.5	-6.8	-6.4
*α*-Amorphene	-6.1	-6.2	-6.3	-6.5	-6.0	-6.1	-6.6	-6.6	-6.2
*α*-Curcumene	-6.3	-6.6	-6.7	-6.5	-6.5	-6.0	-6.8	-6.4	-6.3
*α*-Zingibirene	-5.4	-6.5	-6.4	-6.0	-5.5	-5.6	-5.7	-6.0	-6.2
*α*-Bisabolene	-5.6	-6.8	-6.6	-6.4	-6.4	-5.8	-6.4	-5.9	-6.2
*β*-Sesquiphellandrene	-5.9	-7.0	-7.1	-6.8	6.8	-6.7	-7.1	-6.9	-6.9
Rifamycin SV	-8.7	-9.8	—	-8.7	-8.6	—	-9.6	-10.2	—
Ciprofloxacin	—	—	-7.4	—	—	-6.3	—	—	-6.5

**Table 5:** Interactions details of thymol and *β*-sesquiphellandrene with the selected bacterial targets.

Bacteria	Compound	Targets	Number of Residues Interacting	Residues with H-bond
*S. aureus* ATCC 700699	Thymol	DNA polymerase	4	LYS228
		RNA polymerase	4	—
		Topoisomerase II	6	GLU609, ASP610
	*β*-Sesquiphellandrene	DNA polymerase	1	—
		RNA polymerase	7	—
		Topoisomerase II	8	—
*S. enterica* Typhimurium ATCC 700720	Thymol	DNA polymerase	5	—
		RNA polymerase	1	—
		Topoisomerase II	6	ASN588
	*β*-Sesquiphellandrene	DNA polymerase	8	—
		RNA polymerase	5	—
		Topoisomerase II	6	—
*L. monocytogenes* ATCC 19115	Thymol	DNA polymerase	8	—
		RNA polymerase	5	—
		Topoisomerase II	3	VAL113
	*β*-Sesquiphellandrene	DNA polymerase	6	—
		RNA polymerase	4	—
		Topoisomerase II	5	—

**Table 6:** Toxicity predictions of TVEO compounds using the VEGA QSAR model.

Toxicity measurements	Mutagenicity (Ames Test) Model (CAESAR) 2.1.13	Carcinogenicity model (CAESAR) 2.1.9	Developmental/Reproductive Toxicity Library (PG) 1.1.0	Estrogen receptor relative binding affinity model (IRFMN)	Androgen receptor-mediated effect (IRFMN/COMPARA) 1.0.0	Thyroid receptor alpha effect (NRMEA) 1.0.0	Thyroid receptor beta effect (NRMEA) 1.0.0	In vitro micronucleus activity (IRFMN/VERMEER) 1.0.0
Compound								
*α*-Pinene	Nonmutagenic	Noncarcinogen	Nontoxicant	Inactive	Nonactive	Inactive	Inactive	Inactive
*α*-Thujene	Nonmutagenic	Noncarcinogen	Nontoxicant	Inactive	Nonactive	Inactive	Inactive	Inactive
Camphene	Nonmutagenic	Noncarcinogen	Nontoxicant	Inactive	Nonactive	Inactive	Inactive	Inactive
*β*-Pinene	Nonmutagenic	Noncarcinogen	Nontoxicant	Inactive	Nonactive	Inactive	Inactive	Inactive
*β*-Myrcene	Nonmutagenic	Carcinogen	Nontoxicant	Inactive	Nonactive	Inactive	Inactive	Active
*α*-Fellandrene	Nonmutagenic	Noncarcinogen	Nontoxicant	Inactive	Nonactive	Inactive	Inactive	Active
3-Carene	Nonmutagenic	Noncarcinogen	Nontoxicant	Inactive	Nonactive	Inactive	Inactive	Inactive
D-Limonene	Nonmutagenic	Carcinogen	Nontoxicant	Inactive	Nonactive	Inactive	Inactive	Inactive
O-Cymene	Nonmutagenic	Noncarcinogen	Toxicant	Inactive	Nonactive	Inactive	Inactive	Not predicted
Cymol	Nonmutagenic	Noncarcinogen	Toxicant	Inactive	Nonactive	Inactive	Inactive	Not predicted
*γ*-Terpinene	Nonmutagenic	Noncarcinogen	Nontoxicant	Inactive	Nonactive	Inactive	Inactive	Inactive
Terpinolene	Nonmutagenic	Noncarcinogen	Nontoxicant	Inactive	Nonactive	Inactive	Inactive	Inactive
Linalool	Nonmutagenic	Non carcinogen	Nontoxicant	Inactive	Nonactive	Inactive	Inactive	Inactive
Camphor	Nonmutagenic	Noncarcinogen	Toxicant	Inactive	Nonactive	Inactive	Inactive	Active
Borneol	Nonmutagenic	Noncarcinogen	Nontoxicant	Inactive	Nonactive	Inactive	Inactive	Inactive
4-Terpineol	Nonmutagenic	Noncarcinogen	Nontoxicant	Inactive	Nonactive	Inactive	Inactive	Inactive
*α*-Terpineol	Nonmutagenic	Noncarcinogen	Nontoxicant	Inactive	Nonactive	Inactive	Inactive	Inactive
Thymol methyl ether	Nonmutagenic	Carcinogen	Nontoxicant	Inactive	Nonactive	Inactive	Inactive	Active
Thymol	Nonmutagenic	Noncarcinogen	Nontoxicant	Inactive	Nonactive	Inactive	Inactive	Inactive
Caryophyllene	Nonmutagenic	Carcinogen	Nontoxicant	Inactive	Nonactive	Inactive	Inactive	Inactive
*α*-Humulene	Nonmutagenic	Noncarcinogen	Nontoxicant	Inactive	Nonactive	Inactive	Inactive	Active
*α*-Amorphene	Nonmutagenic	Carcinogen	Nontoxicant	Inactive	Nonactive	Inactive	Inactive	Inactive
*α*-Curcumene	Nonmutagenic	Noncarcinogen	Toxicant	Inactive	Active	Inactive	Inactive	Active
*α*-Zingibirene	Nonmutagenic	Carcinogen	Nontoxicant	Inactive	Nonactive	Inactive	Inactive	Active
*α*-Bisabolene	Nonmutagenic	Noncarcinogen	Nontoxicant	Inactive	Nonactive	Inactive	Inactive	Inactive
*β*-Sesquiphellandrene	Nonmutagenic	Noncarcinogen	Nontoxicant	Inactive	Nonactive	Inactive	Inactive	Inactive
Rifamycin SV	Mutagenic	Noncarcinogen	Nontoxicant	Inactive	Nonactive	Inactive	Inactive	Active
Ciprofloxacin	Mutagenic	Noncarcinogen	Toxicant	Inactive	Nonactive	Inactive	Inactive	Active

**Table 7:** TVEO compounds pharmacokinetic properties prediction using SwissADME.

Compound	Pharmacokinetics								Drug-likeness and Medicinal chemistry				
	GI absorption	BBB permeant	P-gp substrate	CYP1A2 inhibitor	CYP2C9 inhibitor	CYP2D6 inhibitor	CYP3A4 inhibitor	Log K_p__(cm/s)_	Lipinski	Veber	Bioavailability score	PAINS	Synthetic accessibility
*α*-Pinene	Low	Yes	No	No	Yes	No	No	-3.95	Yes	Yes	0.55	0 alert	4.44
*α*-Thujene	Low	Yes	No	No	No	No	No	-5.11	Yes	Yes	0.55	0 alert	3.99
Camphene	Low	Yes	No	No	Yes	No	No	-4.13	Yes	Yes	0.55	0 alert	3.50
*β*-Pinene	Low	Yes	No	No	Yes	No	No	-4.18	Yes	Yes	0.55	0 alert	3.73
*β*-Myrcene	Low	Yes	No	No	No	No	No	-4.17	Yes	Yes	0.55	0 alert	2.85
*α*-Fellandrene	Low	Yes	No	No	No	No	No	-4.85	Yes	Yes	0.55	0 alert	4.15
3-Carene	Low	Yes	No	No	Yes	No	No	-4.02	Yes	Yes	0.55	0 alert	3.84
D-Limonene	Low	Yes	No	No	Yes	No	No	-3.89	Yes	Yes	0.55	0 alert	3.46
O-Cymene	Low	Yes	No	No	No	Yes	No	-4.01	Yes	Yes	0.55	0 alert	1.00
Cymol	Low	Yes	No	No	No	Yes	No	-4.21	Yes	Yes	0.55	0 alert	1.00
*γ*-Terpinene	Low	Yes	No	No	Yes	No	No	-3.94	Yes	Yes	0.55	0 alert	3.11
Terpinolene	Low	Yes	No	No	Yes	No	No	-3.96	Yes	Yes	0.55	0 alert	2.98
Linalool	High	Yes	No	No	No	No	No	-5.13	Yes	Yes	0.55	0 alert	2.74
Camphor	High	Yes	No	No	No	No	No	-5.67	Yes	Yes	0.55	0 alert	3.22
Borneol	High	Yes	No	No	No	No	No	-5.31	Yes	Yes	0.55	0 alert	3.43
4-Terpineol	High	Yes	No	No	No	No	No	-4.93	Yes	Yes	0.55	0 alert	3.28
*α*-Terpineol	High	Yes	No	No	No	No	No	-4.83	Yes	Yes	0.55	0 alert	3.24
Thymol methyl ether	High	Yes	No	Yes	No	Yes	No	-4.64	Yes	Yes	0.55	0 alert	1.09
Thymol	High	Yes	No	Yes	No	No	No	-4.87	Yes	Yes	0.55	0 alert	1.00
Caryophyllene	Low	No	No	No	Yes	No	No	-4.44	Yes	Yes	0.55	0 alert	4.51
*α*-Humulene	Low	No	No	No	Yes	No	No	-4.32	Yes	Yes	0.55	0 alert	3.66
*α*-Amorphene	Low	No	No	No	Yes	No	No	-4.65	Yes	Yes	0.55	0 alert	4.35
*α*-Curcumene	Low	No	No	No	No	Yes	No	-3.71	Yes	Yes	0.55	0 alert	2.31
*α*-Zingibirene	Low	No	No	No	Yes	No	No	-3.88	Yes	Yes	0.55	0 alert	4.81
*α*-Bisabolene	Low	No	No	No	Yes	No	No	-3.03	Yes	Yes	0.55	0 alert	3.90
*β*-Sesquiphellandrene	Low	No	No	No	Yes	No	No	-3.71	Yes	Yes	0.55	0 alert	4.42

**Table 8:** PASS prediction of TVEO compounds activity spectrum.

Compound	Pa	Pi	Possible biological activities
*α*-Pinene	0.821	0.004	Cardiovascular analeptic
	0.746	0.010	Antidyskinetic
	0.706	0.006	Carminative
*α*-Thujene	0.866	0.008	Antieczematic
	0.807	0.006	Anti-inflammatory
	0.729	0.063	Phobic disorder treatment
Camphene	0.882	0.006	Antieczematic
	0.782	0.040	Phobic disorder treatment
	0.738	0.015	Alkylacetylglycerophosphatase inhibitor
*β*-Pinene	0.902	0.005	Antieczematic
	0.735	0.004	Ovulation inhibitor
	0.729	0.013	Respiratory analeptic
*β*-Myrcene	0.941	0.004	Mucomembranous protector
	0.892	0.004	Antineoplastic (breast cancer)
	0.756	0.002	Antiviral (Rhinovirus)
*α*-Fellandrene	0.869	0.012	Ubiquinol-cytochrome c reductase inhibitor
	0.753	0.009	Fibrinolytic
	0.727	0.005	Adenomatous polyposis treatment
3-Carene	0.815	0.005	Antidyskinetic
	0.718	0.034	Antiseborrheic
	0.713	0.004	Transplant rejection treatment
D-Limonene	0.961	0.001	Carminative
	0.743	0.004	Acetylcholine neuromuscular blocking agent
	0.740	0.003	Chemoprotective
O-Cymene	0.924	0.004	Ubiquinol-cytochrome c reductase inhibitor
	0.842	0.010	Mucomembranous protector
	0.778	0.005	Fibrinolytic
Cymol	0.831	0.015	Polyporopepsin inhibitor
	0.822	0.005	Omptin inhibitor
	0.796	0.004	Tpr proteinase (*Porphyromonas gingivalis*) inhibitor
*γ*-Terpinene	0.854	0.009	Antieczematic
	0.803	0.033	Phobic disorders treatment
	0.756	0.023	Sugar-phosphatase inhibitor
Terpinolene	0.927	0.004	Glutamate-5-semialdehyde dehydrogenase inhibitor
	0.848	0.003	Carminative
	0.715	0.014	Venombin AB inhibitor
Linalool	0.913	0.003	Cell adhesion molecule inhibitor
	0.803	0.005	Lipid metabolism regulator
	0.725	0.004	Gastrin inhibitor
Camphor	0.922	0.004	Respiratory analeptic
	0.877	0.006	Antiseborrheic
	0.745	0.002	Pediculicide
Borneol	0.872	0.003	Vasoprotector
	0.822	0.002	Peptidoglycan glycosyltransferase inhibitor
	0.781	0.004	Alopecia treatment
4-Terpineol	0.842	0.019	Ubiquinol-cytochrome c reductase inhibitor
	0.796	0.020	Antiseborrheic
	0.729	0.014	Fibrinolytic
*α*-Terpineol	0.825	0.014	Antieczematic
	0.763	0.023	Alkenylglycerophosphocholine hydrolase inhibitor
	0.750	0.048	Aspulvinone dimethylallyltransferase inhibitor
Thymol methyl ether	0.891	0.005	Mucomembranous protector
	0.790	0.019	Antineurotic
	0.723	0.006	Anesthetic general
Thymol	0.913	0.003	Antiseptic
	0.876	0.004	Membrane permeability inhibitor
	0.830	0.003	APOA1 expression enhancer
Caryophyllene	0.915	0.005	Antineoplastic (lung cancer)
	0.847	0.005	Apoptosis agonist
	0.722	0.002	NF-E2-related factor 2 stimulant
*α*-Humulene	0.818	0.003	MMP9 expression inhibitor
	0.769	0.002	Interleukin agonist
	0.741	0.011	Anti-inflammatory
*α*-Amorphene	0.850	0.003	Carminative
	0.821	0.009	Antineoplastic
	0.726	0.059	Ubiquinol-cytochrome c reductase inhibitor
*α*-Curcumene	0.942	0.004	Mucomembranous protector
	0.757	0.003	Vitamin-K-epoxide reductase (warfarin-insensitive) inhibitor
	0.723	0.003	BRAF expression inhibitor
*α*-Zingibirene	0.842	0.010	Mucomembranous protector
	0.785	0.008	Fibrinolytic
	0.711	0.002	Antiviral (rhinovirus)
*α*-Bisabolene	0.920	0.004	Antieczematic
	0.867	0.003	Carminative
	0.760	0.017	Antineoplastic
*β*-Sesquiphellandrene	0.827	0.009	Antineoplastic
	0.750	0.004	Antipsoriatic
	0.702	0.016	Immunosuppressant

Pa^∗^ represents probability to be active; Pi^∗^ represents probability to be inactive.

## Data Availability

All the relevant data have been provided in the manuscript. The authors will provide additional details if required.
